This article has been retracted.

# Left Ventricular Non-Compaction in Children: Aetiology and Diagnostic Criteria

**DOI:** 10.3390/diagnostics14010115

**Published:** 2024-01-04

**Authors:** Emanuele Monda, Gianantonio De Michele, Gaetano Diana, Federica Verrillo, Marta Rubino, Annapaola Cirillo, Adelaide Fusco, Federica Amodio, Martina Caiazza, Francesca Dongiglio, Giuseppe Palmiero, Pietro Buono, Maria Giovanna Russo, Giuseppe Limongelli

**Affiliations:** 1 Inherited and Rare Cardiovascular Diseases, Department of Translational Medical Sciences, University of Campania “Luigi Vanvitelli”, Monaldi Hospital, 80131 Naples, Italy; emanuelemonda@me.com (E.M.); giandemichele95@gmail.com (G.D.M.); gaetanodiana1991@gmail.com (G.D.); fedeverrillo@gmail.com (F.V.); rubinomarta@libero.it (M.R.); cirilloannapaola@gmail.com (A.C.); adelaidefusco@hotmail.it (A.F.); amodio.federica@yahoo.it (F.A.); martina.caiazza@yahoo.it (M.C.); f.dongiglio@gmail.com (F.D.); g.palmiero@hotmail.it (G.P.); mgiovannarusso@gmail.com (M.G.R.); 2 Institute of Cardiovascular Science, University College London, London WC1N 3JH, UK; 3 Department of Maternal and Child Health, General Directorate for Health, 80131 Naples, Italy; pietro.buono2@regione.campania.it

**Keywords:** left ventricular non-compaction, diagnosis, etiology

## Abstract

Left ventricular non-compaction (LVNC) is a heterogeneous myocardial disorder characterized by prominent trabeculae protruding into the left ventricular lumen and deep intertrabecular recesses. LVNC can manifest in isolation or alongside other heart muscle diseases. Its occurrence among children is rising due to advancements in imaging techniques. The origins of LVNC are diverse, involving both genetic and acquired forms. The clinical manifestation varies greatly, with some cases presenting no symptoms, while others typically manifesting with heart failure, systemic embolism, and arrhythmias. Diagnosis mainly relies on assessing heart structure using imaging tools like echocardiography and cardiac magnetic resonance. However, the absence of a universally agreed-upon standard and limitations in diagnostic criteria have led to ongoing debates in the scientific community regarding the most reliable methods. Further research is crucial to enhance the diagnosis of LVNC, particularly in early life stages.

## 1. Introduction

Left ventricular non-compaction (LVNC), more accurately referred to as left ventricular (LV) hypertrabeculation, as per the recent guidelines by the European Society of Cardiology (ESC) on the management of cardiomyopathies [1], is a heterogeneous myocardial disorder characterized by prominent trabeculae protruding into the LV lumen and deep intertrabecular recesses. The LV myocardium exhibits two distinct layers: compact and non-compact [2]. While the hypertrabecular pattern is primarily observed in the LV, there are cases where the right ventricle (RV) may also be affected, either concurrently with the LV or as an isolated form of the disease [3]. The American Heart Association (AHA) classifies LVNC as a primary cardiomyopathy with a genetic basis [4]. In contrast, in the ESC classification of cardiomyopathies, LVNC falls under the category of “unclassified” cardiomyopathy [5]. In addition, the task force of the recent ESC guidelines on the management of cardiomyopathy does not consider LVNC a cardiomyopathy, but a phenotypic trait that can occur either in isolation or in association with other conditions, such as LV hypertrophy, dilatation, systolic dysfunction, or developmental abnormalities [1].

The substantial diversity in the clinical presentations of hearts meeting the diagnostic criteria for LVNC, the existence of multiple conditions where diagnostic criteria are met despite normal systolic and diastolic function, and scenarios where the hypertrabecular pattern appears reversibly create challenges for clinicians in distinguishing between cardiomyopathy and a variation of the normal LV anatomy. This necessitates caution in the application of diagnostic criteria, particularly in patients displaying no symptoms and lacking a family history of cardiomyopathy. Furthermore, although echocardiography and cardiac magnetic resonance (CMR) imaging are the basis for the diagnostic criteria [6], there is no universally accepted gold standard for the diagnosis of LVNC.

This review aims to provide an overview of the literature concerning the clinical and genetic characteristics of LVNC and to explore the role of the proposed diagnostic criteria.

## 2. Prevalence

Large-scale studies using echocardiography in both children and adults have estimated the prevalence of so-called non-compaction cardiomyopathy to be between 0.02% and 0.14% [7,8,9,10].

In the pediatric age group, the number of reported LVNC cases has been increasing over the last few decades, possibly not due to an actual increase in cases but rather because of the improved accuracy of imaging methods [11]. Among children, LVNC ranks as the third most prevalent cardiomyopathy after dilated cardiomyopathy (DCM) and hypertrophic cardiomyopathy (HCM) [12]. Cases of LVNC have been reported at various ages, including neonates [13] and during the prenatal period [14]. Between 2004 and 2013, Tian et al. [14] documented nine cases of LVNC in fetal echocardiography using the criteria proposed by Jenni [15] and Stollemberg [16]. At birth, LVNC was confirmed in two cases via echocardiography, while the remaining seven pregnancies were terminated, with diagnosis was confirmed during autopsy.

The incidence of LVNC has been estimated at 0.12 per 100,000 in children up to 10 years of age and 0.81 per 100,000 in children up to one year of age [17]. Furthermore, a large registry encompassing 98 centers in the USA and Canada over an 18-year span revealed that 4.8% of pediatric cardiomyopathies corresponded to LVNC [18]. In most LVNC cases, there was an association with other cardiomyopathies (59% with DCM and 11% with HCM), while 23% presented as an isolated phenotype and 8% as an indeterminate phenotype [18]. The age of onset was higher for isolated forms of LVNC (average 9.8 years) compared to those associated with other cardiomyopathies (0.4–0.6 years) [18]. From April 2016 to October 2018 in Denmark, Borresen et al. [13] conducted echocardiograms on 21,133 healthy infants revealing an LVNC prevalence of 0.076%. LVNC was defined on the echocardiogram by the ratio of non-compact (NC) to compact (C) layers thicknesses (NC/C ≥ 2) in end-diastole. However, the absence of a universally accepted gold standard for diagnosing LVNC renders the incidence and prevalence of this cardiomyopathy uncertain.

## 3. Pathogenesis

The prevailing pathogenetic hypothesis for the development of LVNC is the myocardium non-compaction hypothesis. During the fourth week of gestation, the epicardium and the coronary artery system have not yet fully developed. At this stage, nourishing the cardiac cells necessitates a large exchange surface to facilitate the diffusion of nutrients and oxygen from the blood through the endocardial layer [19]. This is achieved through the formation of a network of myocardial trabeculae and deep intertrabecular recesses, which significantly increase the available surface area for exchange [19].

Consequently, the myocardium is divided into two layers: the first, subepicardial, being the “compact” layer, and the second, thicker layer referred to as “non-compact”. Between the fifth and eighth weeks of gestation, the epicardium covers the myocardium, marking the development of the coronary circulation and the transition from nourishment through diffusion to active circulation, as seen in adults. During this period, compaction of the myocardium takes place, proceeding from the base to the apex [20] and from the epicardium to the endocardium. This results in the reduction in the NC/C ratio. Anomalies in this process were initially considered as a potential explanation for the development of LVNC.

Simultaneously, both the trabecular and compact myocardial layer experience significant growth during development, though not always in equal proportions [21]. The thickness ratio between these layers decreases during development, despite an increase in the volume of both layers, indicating greater growth in the compact layer compared to the trabecular layer. Pulse labelling and immunohistochemical studies further support these morphometric observations, showing a greater proliferation of cardiomyocytes in the compact wall compared to the layers the trabeculations [22,23,24]. When proliferation is experimentally inhibited in the trabecular layer, the compact mural thickness remains largely unaffected [14]. Luxan et al. [23] also demonstrated that in mice with inactivation of the *MIB1* gene (known to induce LVNC in humans), LVNC developed due to proliferation (10–15%) of the non-compact myocardium.

The compact wall can develop normally even when excessive trabeculation is induced via the suppression of NKX2-5 [25]. This suggests that the growth of the compact wall is largely independent of that in the trabecular layer. Contrary to earlier notions suggesting that the compact layer forms as a result of the compaction of pre-existing trabeculations, contemporary observations indicate continuous positive growth of the trabecular and compact myocardial layers. This evidence implies that the hypertrabecular phenotype arises from a thickening of the non-compact layer rather than a failure to compact. Therefore, it is recommended to use the term LV hypertrabeculation rather than LVNC. In addition, the concept of intrauterine arrest in the process of compaction has been suggested but lacks supporting evidence [26,27]. Consequently, the term non-compaction has no basis in myocardial development [28,29,30].

Next to the cases of LVNC presenting during the neonatal period, there are different scenarios where LVNC can be an acquired phenotype. It has been suggested that increased hemodynamic load on the LV, such as pregnancy or physical activity, may lead to the development of LVNC. For example, Paun et al. [31] showed that the appearance of trabeculations on the LV wall can be considered an adaptive response to meet the increased hemodynamic demands of the individuals, demonstrating a relationship between the increase in trabeculations and the increase in stroke volume.

## 4. Etiology

LVNC can manifest as either a sporadic or familial disease. According to an ESC position statement [5], cardiomyopathies can be classified into familial/genetic or non-familial/non-genetic forms [4]. Familial forms are defined as those in which the same phenotype, or one caused by the same mutation, occurs in more than one member. This also includes cases occurring in a single family member but driven by a de novo mutation that may be inherited by their offspring. Additionally, genetic forms of LVNC encompass cases in which LVNC is a cardiac manifestation of a multi-organ disease, such as tafazzinopathies. In contrast, sporadic cardiomyopathy refers to cases of LVNC that do not occur in other relatives. Sporadic forms of LVNC include idiopathic forms, where no identifiable cause is found, or acquired forms, such as those resulting from increased hemodynamic load on the LV.

For familial cases, the primary mode of transmission is typically autosomal dominant [32,33], followed by X-linked transmission, while autosomal recessive transmission is less common [32]. Family pedigrees often show variable penetrance in LVNC transmission [34]. Moreover, it has been observed that within a single family, a genetic mutation responsible for LVNC may be associated with phenotypic heterogeneity and varying ages of onset [34]. When a new case of LVNC is identified, clinical and echocardiographic screening of family members is recommended to detect cardiomyopathy in relatives and to identify family members at risk of developing LVNC.

There are currently no established guidelines for genetic testing in patients with LVNC. However, a consensus statement by the Heart Rhythm Society (HRS) and the European Heart Rhythm Association (EHRA) suggests that genetic testing may be considered for patients diagnosed with LVNC, except in cases where the diagnosis of LVNC is incidental, without symptoms, family history, or associated syndromes [35]. It is important to note that the positivity rate of genetic testing is low in patients with LVNC who lack systolic dysfunction, a family history, or associated syndromes. Approximately 17% and 50% of cases [36] reveal the genetic mutation responsible for LVNC. A retrospective study conducted in the Netherlands [36] demonstrated that in the pediatric age group, the yield of genetic testing was higher than in adults (45% vs. 30%).

### 4.1. Genetic Forms of LVNC

Genetic variability in LVNC, like in other cardiomyopathies, is known to be exceptionally high. However, data on genetic mutations responsible for LVNC in pediatric cases are limited, primarily due to the relatively low rate of genetic testing conducted in children. The genes associated with LVNC are reported in Table 1.

The *TAZ* gene, which encodes for the protein tafazzin, was the first gene discovered to be linked to LVNC [37]. Mutations in this gene are responsible for Barth syndrome, which is a X-linked disease characterized by neutropenia, myopathy, and cardiomyopathy [38]. Recent studies involving the silencing of *TAZ* in mice provide valuable insights into understanding the cardiomyopathy associated with Barth syndrome and offer a platform for testing potential therapeutic approaches [39].

LVNC has been described in conjunction with other syndromes, including dystrophinopathies (such as Duchenne and Becker muscular dystrophy), Charcot–Marie–Tooth syndrome 1A, mitochondrial diseases, and various syndromes such as Turner, DiGeorge, Melnick–Needles, nail–patella, Noonan, and Beals syndromes [6].

An examination of CMR scans in a substantial group of individuals with Duchenne muscular dystrophy found that about 30% of patients displayed excessive trabeculation in at least one cardiac segment according to the Petersen diagnostic criteria [40,41]. Follow-up studies carried out on a subset of Duchenne muscular dystrophy patients reported an annual rate of change in the NC/C ratio of +0.4 [41]. This alteration was linked to a gradual increase in the thickness of the trabecular layer alongside a simultaneous reduction in the thickness of the compact wall. These findings led investigators to propose that Duchenne cardiomyopathy represents a progressive disease marked by a fragile cytoskeleton, ultimately resulting in the deterioration of LV systolic function and compensatory remodeling of the trabecular myocardium over time [41,42].

Various other genes have been associated with LVNC, such as those encoding for sarcomeric proteins. However, the precise mechanism through which pathogenic mutations in these genes lead to LVNC remain largely unknown. *MYH7* (encoding for beta myosin heavy chain) and *MYBPC3* (encoding for myosin chain binding protein C) are the most commonly sarcomeric genes associated with LVNC, accounting for approximately 25% and 10% of cases, respectively [43]. Mutations in the *TTN* gene, encoding for titin, should also be acknowledged as a cause of LVNC. Other pathogenic mutations are described in genes encoding for desmosomal proteins [44]. Parent et al. [45] described LVNC in patients with mutations of *LMNA*, a gene synthesizing components of the nuclear membrane, which typically leads to DCM with conduction disturbances. Pathogenic mutations in *LDB3* have also been described. This gene is involved in the synthesis of Z-lineage components in both cardiac and skeletal muscle, and associated mutations have been associated with DCM, LVNC, and overlapping conditions [46]. Furthermore, while the *ZASP1* p.D117N variant has been described in a patient with LVNC and conduction disorders [47], Levitas et al. [48] suggested that the role of this mutation in heart disease requires further evaluation.

Pathogenetic mutations in the *SCN5A* gene, which encodes for the alpha subunit of the cardiac sodium channel, have been observed in LVNC cases [6]. Carriers of specific pathogenetic mutations in this gene are at an elevated risk of arrhythmias and a higher likelihood of heart failure progression [49]. Moreover, mutations in potassium channel genes have also been associated with LVNC, sometimes accompanied by prolonged QT intervals [50,51]. Other associations include LVNC with atrial fibrillation [52] and catecholaminergic polymorphic ventricular tachycardia [53].

An association between LVNC and congenital heart diseases, such as LV and/or right ventricular outflow tract obstructions, bicuspid or unicuspid aortic valve, aortic coarctation, Ebstein anomaly, tetralogy of Fallot, and double outlet right ventricle has also been documented [54]. Furthermore, a genetic relationship between Ebstein anomaly and right ventricular non-compaction has been described in individuals with *MYH7* mutation [55].

Given the considerable genetic heterogeneity in LVNC, some authors [56] suggest conducting a comprehensive genetic analysis rather than restricting the analysis of only those genes known to cause LVNC. Current guidelines recommend genetic testing based on the presence of features suggestive for other associated cardiomyopathy [57], rather than conducting genetic testing when the phenotypic feature of excessive trabeculation is incidentally detected in patients who are asymptomatic and have otherwise normal cardiac findings.

### 4.2. Non-Genetic/Acquired Forms of LVNC

LVNC can manifest as a sporadic abnormality in response to LV mechanical overload conditions. This is evident in cases involving highly trained athletes, especially those of African/Afro-Caribbean origin, who meet the criteria for LVNC. However, only a small number of them experience a reduction in systolic function, and none exhibit abnormalities in diastolic function [58]. The prevalence of individuals meeting the criteria for excessive trabeculation, as assessed via echocardiography, in competitive athletes varies between 1.4% and 8.1%. This variation is influenced by different definitions, ethnicities, and specific sports disciplines [59,60].

A study conducted by Gati et al. [59] demonstrated that among 102 primigravid pregnant women, 25% developed LV trabeculations, and eight women met the echocardiographic criteria from Chin et al. [26] and Jenni et al. [15] for the diagnosis of LVNC. Of these women, 69.2% exhibited the disappearance of LV trabeculae in the postnatal period, while an additional 12.8% experienced the disappearance of LV trabeculae occurred over a 24-month follow-up period.

There are cases where the LVNC phenotype appears in the absence of symptoms, LV systolic dysfunction, or dilatation evident on echocardiography. These findings suggest that these instances are not a manifestation of cardiomyopathy but rather a response of the LV myocardium to increased mechanical load, including volume and pressure overload, in predisposed individuals [59]. It is worth noting that African American women were three times more likely to develop such features during pregnancy than Caucasian women [61], hinting at a potential underlying genetic susceptibility in the adaptive response of the myocardium [62].

Cardiac dysfunction related to chemotherapy is now acknowledged as potentially associated with excessive LV trabeculation [63,64]. It was suggested that this phenotype can be the myocardial response to drug toxicity. However, it could be the result, rather than the cause, of cardiac dysfunction. At the same time, even in patients with hemoglobinopathies, excessive trabeculation can be interpreted as the adaptive response to heightened cardiac preload [65].

Several reports have suggested a potential connection between polycystic kidney disease and a cardiomyopathy associated with excessive trabeculation [66,67]. However, it remains uncertain whether this association can be attributed to a genetic interaction between the genes responsible for polycystic kidney disease and those altered in genetic cardiomyopathies [66]. Another explanation could be that excessive trabeculation develops or becomes apparent due to the increased cardiac preload associated with chronic kidney disease.

## 5. Clinical Manifestations

In childhood, as in adulthood, the clinical manifestations of LVNC are highly diverse. The primary clinical presentations encompass heart failure, arrhythmias, and thromboembolic events, either individually or in various combinations [2]. In some cases, LVNC is also diagnosed in asymptomatic patients. At the onset of LVNC, the most common manifestation is heart failure, occurring in 46% of cases, followed by diagnosis in asymptomatic patients or as part of family screening, which accounts for 35% of cases [68].

LVNC can present in isolation or be associated with ventricular systolic or diastolic dysfunction [34]. In hearts that are otherwise normal, the capillarization and the density of sarcomeres and mitochondria are similar in both non-compacted and compact myocardium [69]. Although reproducing the exact anatomy of the trabecular meshwork is a complex task, modeling of LV function has indicated a positive influence of trabeculation on pump function [70]. However, several human studies showed that there is not a significant correlation between the extent of trabecular myocardium and cardiac function [70,71].

Another common feature of LVNC is the development of arrhythmias. Arrhythmias and electrocardiographic abnormalities are more common in patients experiencing heart failure or LV systolic dysfunction [72]. Although the myocardial architecture of excessive trabeculation might seem linked to a predisposition for reentrant tachycardias, there is no evidence supporting this hypothesis. After accounting for confounding factors (e.g., LV dilation, systolic dysfunction, myocardial fibrosis), excessive trabeculation does not appear to be associated with an increased risk of arrhythmias [73]. Ventricular premature ectopias and ventricular tachycardia observed in patients with excessive trabeculation often originate from segments replaced with myocardial scar or from the ventricular outflow tract [74,75].

Abnormal ECGs are also common in pediatric patients with LVNC. However, these ECG abnormalities are nonspecific for LVNC. A study by Brescia et al. [76] showed that the most frequent abnormalities were increased voltages due to left ventricular hypertrophy. Other common findings included repolarization alterations, such as ST-T changes or T-wave inversions. In children, the prevalence of ventricular tachycardias ranged between 0% and 38%, and supraventricular tachycardia occurred between 8% and 13%, with a particular prevalence of atrioventricular re-entry tachycardias or focal atrial tachycardia [34,76]. In the same pediatric cohorts, sudden cardiac death had a prevalence ranging from 0% to 13%, with none occurring in children without previous arrhythmias or those with normal cardiac size and function.

The third major clinical aspect of LVNC is thromboembolism (TE). In childhood, an independent predictor of TE is an LV ejection fraction below 40%. Several reports have documented the presence of LV thrombi in the context of the trabeculations [26]. However, cohort studies do not indicate an increased risk of adverse events in the context of excessive trabeculation, especially in patients with normal LV ejection fraction [77,78,79,80].

## 6. Diagnostic Criteria

In both adult and pediatric age groups, the diagnosis of LVNC relies on morphological criteria. Echocardiography serves as the primary method and is also valuable for patient follow-up. CMR, on the other hand, is a secondary diagnostic tool that aids in confirming the diagnosis and provides prognostic insights by detecting late gadolinium enhancement (LGE).

## 7. Echocardiogram

Due to the lack of a gold standard for the diagnosis of LVNC, various morphological criteria have been proposed, although not all of them have been validated (Figure 1).

In pediatric cases, multiple criteria are available. The most important are summarized in Table 2 and shown in Figure 2.

The criteria published by Jenni et al. are the most commonly used in clinical practice [15]. These criteria include the NC/C ratio (i.e., the ratio of trabecular to compact myocardium) exceeding 2:1, measured in end-systole in the short-axis view. The most pronounced trabeculation is usually observed in the mid-lateral, apical, and mid-inferior segments, and the presumption is the absence of coexisting cardiac abnormalities.

Among 21,133 newborns (average age 11 days) who underwent an echocardiogram using diagnostic criteria for LVNC, the presence of an NC/C ratio > 2 in end-diastole in at least one of the 12 segments of the LV (6 in the apical 4-chamber projection and 6 in the parasternal short-axis projection at the level of the papillary muscles), the segment in which the ratio was most frequently >2 was the apex of the LV, followed by the middle interventricular septum and the middle lateral wall of the LV [13].

While Jenni’s criteria [15] are the most commonly used in clinical practice, Joong et al. [81] demonstrated, in a pediatric population, that the X/Y ratio (the ratio between the distance between the epicardial surface and the bottom of the recesses (X) and the distance between the epicardial surface and the apex of the trabeculae (Y)) measured in the parasternal short axis in the anterolateral apical region at the end of diastole has the highest sensitivity and specificity for diagnosing LVNC. In contrast, the NC/C ratio has the lowest reproducibility and diagnostic validity.

Although based on an adult population, the results of Kohli’s study [82] on a cohort of patients with systolic dysfunction raise some doubts about the specificity of the most widely used morphological ultrasound criteria of LVNC, as 23.6% of those enrolled fulfilled at least one of these criteria, especially among those of African ethnicity. The challenge in accurately identifying the non-compact myocardial border and the limited number of patients in studies used to derive the primary morphological criteria are additional limitations in accurately diagnosing LVNC.

When the LV chamber is challenging to visualize, an echocardiogram with contrast injection or three-dimensional echocardiography can be valuable. The benefits of contrast administration include better visualization of recesses between the trabeculae, improved examination of the flow between them, and enhanced identification of the endocardial border, particularly in the apical region of the ventricle [83].

In speckle tracking echocardiography (STE), a reduction in myocardial strain has been observed in children with LVNC and normal ejection fraction when compared to controls [81]. STE can serve as a method to identify subclinical left ventricular dysfunction in pediatric patients with LVNC, as it detects reductions before conventional echocardiographic methods. Additionally, McMahon et al. [84] demonstrated a decrease in diastolic tissue Doppler velocity in 56 children with LVNC compared to controls.

## 8. Cardiac Magnetic Resonance

Cardiac magnetic resonance (CMR) is typically considered a secondary diagnostic method [84,85,86], providing enhanced visualization of anatomical details, particularly in patients with challenging acoustic chest windows (Figure 3). The primary diagnostic criteria used for the diagnosis of VSNC in adulthood are summarized in Table 3. However, there are currently no dedicated studies of pediatric diagnosis.

In 2005, Petersen et al. [30] described a morphological criterion based on the ratio of the thickness of the two cardiac layers (NC/C). A ratio greater than 2.3 is considered diagnostic. In 2012, the results of the MESA (MultiEthnic Study of Atherosclerosis) [40] revealed that 43% (140 of 323) of the participants had an NC/C ratio exceeding 2.3 at MRI in at least one cardiac region, with 6% having a ratio exceeding 2.3 in more than two cardiac regions. This underscores the need for greater specificity in the diagnostic criterion.

In CMR analysis, Jacqueir et al. [75] based the LVNC diagnosis on the ratio between the trabeculated left ventricular mass and the total mass at the end of diastole.

Captur et al. [85] employed fractal analysis of the endocardial border using automated software for LVNC diagnosis. The presence of numerous trabeculations in LVNC patients results in an irregular endocardial border. Consequently, the fractal dimension (FD), a measure of how fully a complex structure occupies space, is typically increased in patients with LVNC. Specifically, the diagnostic threshold is set at an FD of ≥1.3 in all cardiac segments, except for the apical segment where the threshold is ≥1.26.

Finally, Stacey et al. [86] revealed that an NC/C ratio exceeding 2 at the end of systole showed a stronger correlation with heart failure and adverse events compared to both NC/C at the end of diastole and the ratio of trabecular ventricle mass to the total left ventricle mass.

## 9. Outcome and Prognosis

Multiple studies have identified LV dysfunction as the primary factor influencing adverse outcomes in the presence of excessive trabeculation [73,78]. Individuals with reduced ejection fraction exhibited cardiovascular mortality rates twice as high as those with preserved LV function. Prognostic insights are provided by CMR studies using late gadolinium enhancement (LGE). A meta-analysis including patients with excessive LV trabeculation revealed an increased risk of cardiac events in those with late gadolinium enhancement [77]. An observational study indicated a higher rates of cardiovascular events in patients with excessive trabeculation compared to age-matched patients with dilated cardiomyopathy [89]. However, in another study that underwent multivariable adjustment over a median follow-up period of 5 years, no difference in event-free survival rates was found between dilated cardiomyopathy and cardiomyopathy with excessive trabeculation [90].

In individuals who are otherwise healthy, the phenotypic feature of excessive trabeculation does not appear to have independent prognostic significance. In contrast, in patients with excessive trabeculation and an associated cardiomyopathy phenotype, the risk for adverse events seems to be associated with the latter and appears independent of the coexisting trabeculation.

The prognosis of LVNC in pediatric age is variable and depends on several factors. A study conducted by Brescia et al. [76] highlighted several risk factors for death and cardiac transplantation in pediatric patients with LVNC. Significant risk factors included cardiac dysfunction, with a 5-year survival rate of 98% in subjects with normal cardiac function versus 60% in patients with systolic dysfunction. Another significant predictor of the risk of cardiac death and transplantation was the cardiomyopathy phenotype. At 5 years of follow-up, the survival rate from death and transplantation was 98% in patients with a phenotype associated with normal heart geometry, 86% for the hypertrophic phenotype, 64% for the mixed phenotype, and 63% for the dilated phenotype [91]. Similar results were described by Jefferies et al. [18], with the best outcome for children with isolated LVNC. Other risk factors described in the pediatric cohort of Brescia et al. [76] are ECG abnormalities (T-wave inversion and ST-tract abnormalities) and arrhythmias. Presentation before the age of 1, the association between ventricular arrhythmias and early disease onset are other significant risk factors in the pediatric population for death or transplantation [18,76]. McMahon et al. [84] indicated that a reduced mitral lateral velocity (Ea), measured via echocardiography, has been the most sensitive parameter for identifying children with LVNC at an increased risk of death or the need for cardiac transplantation. Finally, cardiac fibrosis detected with CMR via LGE may be a prognostic factor.

## 10. Anticoagulation

As mentioned before, patients with LVNC present a higher rate of TE. The likelihood of experiencing TEs seems to be age-related, with adults showing an increased risk compared with children [2]. The cause of TEs in children with LVNC is mostly cardio-embolic with significant implications in terms of treatment. However, due to the lack of large studies exploring the efficacy and safety of prophylactic anticoagulant therapy, the choice should be based on the presence of risk factors. The most important factors associated with increase TEs are represented by previous TEs, evidence of cardiac thrombus, or atrial fibrillation [16,80,81]. Another important risk factor is represented by left ventricular systolic dysfunction, and in patients showing this clinical feature, prophylactic therapy may be considered. More debated is the assessment of TE risk in patients with normal LV ejection fraction and without atrial fibrillation and previous TEs. In this scenario, prophylactic therapy should be avoided.

## 11. Conclusions

LVNC is a cardiac condition that may occur in isolation or in association with other cardiomyopathies. In pediatric age, its prevalence is increasing, thanks to improved imaging methods. The etiology of LVNC is highly heterogeneous, encompassing both genetic and acquired forms of the disease. The clinical presentation of LVNC varies widely, and while it can be diagnosed in asymptomatic patients, the most common clinical scenario involves a combination of heart failure, thromboembolism, and arrhythmias. The diagnosis of LVNC primarily relies on morphological assessments through imaging methods such as echocardiography and CMR. However, the absence of a universally accepted “gold standard” and the limitations of some diagnostic criteria in specific patient cohorts have sustained ongoing scientific debates regarding the most reliable morphological diagnostic criteria. Further research is required to refine the diagnosis of LVNC, particularly in the early stages of life.

## Figures and Tables

**Figure 1:** Echocardiographic images of a patient with LVNC. On the (**left**), apical 4-chamber view; on the (**right**), parasternal short-axis view.

**Figure 2:** Comparison of the echocardiographic diagnostic criteria for children with LVNC [7,13,15,26].

**Figure 3:** Cardiac magnetic resonance image of a patient with LVNC.

**Table 1:** Genes associated with left ventricular non-compaction with definitive or moderate evidence, according to Clinical Genome Resource (ClinGen). Abbreviations: AD, autosomal dominant; AR, autosomal recessive; ARVC, arrhythmogenic right ventricular cardiomyopathy; DCM, dilated cardiomyopathy; HCM, hypertrophic cardiomyopathy; RCM, restrictive cardiomyopathy; XL, X-linked.

Gene	Protein	Other Cardiac Phenotypes	Inheritance
**Cytoskeleton**			
*DES*	Desmin	HCM, DCM, ARVC, RCM	AD, AR
*LDB3*	LIM domain binding 3	HCM	AD
*LMNA*	Lamin A/C	DCM	AD, AR
*MIB1*	Mindbomb E3 ubiquitin protein ligase 1	-	AD
**Desmosome**			
*DSP*	Desmoplakin	DCM, ARVC, RCM	AD, AR
*PKP2*	Plakophillin 2	ARVC	AD, AR
**Ion channels and calcium-handling proteins**			
*HCN4*	Hyperpolarization activated cyclic nucleotide-gated potassium channel 4	-	AD
*PLN*	Phospholamban	HCM, DCM, ARVC	AD, AR
*RYR2*	Ryanodine receptor 2	-	AD
*SCN5A*	Sodium channel, voltage-gated, type V, alpha subunit	DCM	AD, AR
**Lysosome**			
*LAMP2*	Lysosome-associated membrane protein 2	HCM	XL
**Mitochondria**			
*NNT*	Nicotinamide nucleotide transhydrogenase	-	AD
*TMEM70*	Transmembrane protein 70	-	AR
**Sarcolemma**			
*DMD*	Dystrophin	DCM	XL
*DMPK*	Dystrophia myotonica-protein kinase	-	AD, AR
*DTNA*	Dystrobrevin alpha	-	AD
**Sarcomere**			
*ACTC1*	Actin alpha cardiac muscle 1	HCM, DCM, RCM	AD
*MYBPC3*	Myosin binding protein C	HCM, RCM	AD, AR
*MYH7*	Myosin beta heavy chain 7	HCM, DCM, RCM	AD, AR
*TNNT2*	Troponin T type 2	HCM, DCM, RCM	AD
*TPM1*	Alpha tropomyosin 1	HCM, DCM, RCM	AD
*TTN*	Titin	HCM, DCM, RCM	AD, AR
**Signal Transduction and Trascriptional Factors**			
*ALPK3*	Alpha kinase 3	HCM	AD
*NKX2-5*	NK2 homeobox 5	-	AD
*NONO*	Non-POU domain containing octamer binding protein	-	AD
*PRMD16*	PR domain containing 16	-	AD
*RBM20*	RNA binding motif protein 20	DCM	AD
*TAZ*	Tafazzin	-	XL
*TBX5*	T-box 5	-	AD
*TBX20*	T-box 20	-	AD

**Table 2:** Proposed echocardiographic criteria for the diagnosis of left ventricular non-compaction in children.

Name	Chin et al. [26]	Jenni et al. [15]	Børresen et al. [13]	Pignatelli et al. [7]
Patients (n)	8	34	16	36
Age	0.9–22.5 years	16–75 years	7–15 days	1–15 years
Criteria description	Ratio of the distance between the epicardial surface and the bottom of the recesses (X) to the distance between the epicardial surface and the apex of the trabeculae (Y)	Absence of a coexisting cardiac abnormality Appearance of numerous prominent trabeculations with deep intertrabecular recesses Intertrabecular spaces filled with blood, visualized on color Doppler imaging Non-compact/compact ratio at the site of maximum myocardial wall thickness	Thickness ratio between non-compact and compact layer of the left ventricle wall in at least 1 of the 12 cardiac segments assessed	Presence of multiple trabeculations Multiple intertrabecular recesses communicating with the ventricular cavity, visible on color Doppler imaging Ratio of the thickness of the non-compact layer to the compact layer of the LV wall (NC/C)
Cardiac cycle	End-diastole	End-systole	End-diastole	End-systole
Echocardiographic projection recommended	Apical 4-chamber view Parasternal long-axis view	Parasternal short-axis view	6 segments in the apical 4-chamber view 6 segments in the parasternal short axis view at papillary muscle level	Parasternal short axis view
**Ratio**	X/Y ≤ 0.5	NC/C ratio > 2	NC/C ratio > 2	NC/C ratio > 1.5

**Table 3:** Proposed cardiac magnetic resonance criteria for the diagnosis of LVNC in adults. Abbreviations: LV, left ventricular.

Name	Petersen et al. [30]	Jacquier et al. [75]	Stacey et al. [86]	Grothoff et al. [87]	Captur et al. [85]	Choi et al. [88]
**Patients (n)**	7	16	122	12	30	145
Age	14–46 years	31–65 years	42–72 years	11–51 years	28–54 years	39–74 years
**Criteria description**	The ratio between the thickness of the non-compact and compact layer	Percentage of trabeculated LV mass compared to overall LV mass	Ratio between the thickness of the non-compact and compact layer	Percentage of non-compact LV mass Total mass of non-compact LV NC/C (excluding segment 17)	Highest fractal dimension (FD)	Percentage of LV trabecular volume in relation to overall LV volume
**Cardiac cycle**	End-diastole	End-diastole	End-systole	End-diastole	End-diastole	End-diastole
**Projection recommended**	Parasternal long-axis view	Parasternal short-axis view	Parasternal short-axis view	Parasternal short-axis view	Parasternal short-axis view	Parasternal short-axis view
**Ratio**	NC/C > 2.3	LV trabeculated mass > 20%	NC/C > 2	>25% of left ventricular mass noncompact >15 g/m^2^ of the total noncompact mass of the left ventricle NC/C > 2 or >3 depending on the segments considered	Global highest FD ≥ 1.26; Apical highest FD ≥ 1.3	LV trabeculated volume > 35%

## Data Availability

Not applicable.
